# Genome Sequences of Five SARS-CoV-2 Variants from Mumbai, India, Obtained by Nanopore Sequencing

**DOI:** 10.1128/MRA.00231-21

**Published:** 2021-04-15

**Authors:** Kayzad Nilgiriwala, Ayan Mandal, Grishma Patel, Tejal Mestry, Smriti Vaswani, Ambreen Shaikh, Kalpana Sriraman, Swapneil Parikh, Shreevatsa Udupa, Nirjhar Chatterjee, Jayanthi Shastri, Nerges Mistry

**Affiliations:** a The Foundation for Medical Research, Worli, Mumbai, India; b Kasturba Hospital, Arya Nagar, Chinchpokli, Mumbai, Maharashtra, India; DOE Joint Genome Institute

## Abstract

We report here the genome sequences of severe acute respiratory syndrome coronavirus 2 (SARS-CoV-2) variants from five coronavirus disease 2019 (COVID-19) patients in Mumbai, India. Viral genomic RNA was isolated from nasopharyngeal swabs and/or respiratory particles from the masks of the patients. Genomic variant analysis determined 8 to 22 mutations, and the variants belong to lineages previously associated with Indian variants.

## Abstract (precis)

We report here the genome sequences of SARS-CoV-2 variants from five COVID-19 patients in Mumbai, India. Viral genomic RNA was isolated from nasopharyngeal swabs and/or respiratory particles from the masks of the patients. Genomic variant analysis determined 8 to 22 mutations, and the variants belong to lineages previously associated with Indian variants.

## ANNOUNCEMENT

With an increasing rate of infection that has reached nearly 122 million globally and 11.5 million in India as of 18 March 2021, the coronavirus disease 2019 (COVID-19) pandemic has grown dramatically over a span of 1 year. The genome sequences of severe acute respiratory syndrome coronavirus 2 (SARS-CoV-2) (family *Coronaviridae*, genus *Betacoronavirus*) help us to provide insights for fighting against the disease, which has so far been estimated to cause 2.06 million deaths worldwide (https://covid19.who.int/).

In this study, we present the genome sequence of SARS-CoV-2 viruses from five COVID-19 patients, collected between August and September 2020 from Kasturba Hospital for Infectious Diseases in Mumbai, India. The study was undertaken between June and September 2020 after approval by the Institutional Research Ethics Committee of the Foundation for Medical Research (FMR), Mumbai (FMR/IREC/TB/01/2020), and the Institutional Review Board of Kasturba Hospital for Infectious Diseases (IRB-09/2020). Four out of the five samples were obtained from nasopharyngeal swabs (NPS), whereas one sample (CMP-19/2020) was obtained from a modified N-95 mask worn by the patient (1). The patients ranged in age from 17 to 68 years old and had presented with mild to moderate symptoms of COVID-19, including fever, cough, and weakness, with their cycle threshold (*C_T_*) values ranging from 20 to 31. The RNA from NPS was extracted using the MagMax viral/pathogenic nucleic acid isolation kit via the KingFisher Flex system (Thermo Fisher Scientific, USA), while the RNA from the mask was extracted using the QIAamp viral RNA minikit (Qiagen, Germany) as per a protocol used earlier (1). The cDNA was synthesized using the high-capacity cDNA reverse transcription kit (Thermo Fisher Scientific).

Whole-genome sequencing was conducted using the ARTIC amplicon sequencing protocol (2) and GridION sequencer (Oxford Nanopore Technologies, UK). Base calling was performed using Guppy v3.5.1 in high accuracy mode (3). The processed reads were subjected to filtering using the fieldbioinformatics v1.1.3 pipeline (https://github.com/artic-network/fieldbioinformatics). The variants identified were further annotated using SnpEff v4.3 (4). A range of 8 to 22 mutations were observed in the genome sequences of the five variants (Table 1). All five variants had the D614G mutation in the spike protein (5) and c14408t in the *ORF1ab* gene. All tools were run with default parameters unless otherwise specified.

**TABLE 1:** Nucleotide and amino acid changes in all five strains in comparison to the Wuhan-Hu-1 reference strain (GenBank accession number MN908947.3)

Characteristic					Data for strain^*a*^:				
					India/MH-CMP-19/2020	India/MH-CMP-30/2020	India/MH-CMP-31/2020	India/MH-CMP-34/2020	India/MH-CMP-35/2020
GenBank accession no.					MW645473	MW645474	MW645475	MW645476	MW645477
SRA accession no.					SRR13892481	SRR13892480	SRR13892479	SRR13892478	SRR13892477
Genome size (no. of base pairs)					29,694	29,866	29,696	29,866	29,866
Genome coverage (%)					99.30	99.88	99.31	99.88	99.88
GC content (%)					39	40	39	38	39
Variants in the sequences				
Position	Reference	Variant	Gene	Amino acid change
241	C	T			*		*	*
313	C	T	*ORF1ab*			*		*	*
455	C	T	*ORF1ab*	L64F			*		
1642	C	T	*ORF1ab*					*	
1823	G	A	*ORF1ab*	A520T			*		
1957	G	A	*ORF1ab*					*	
3037	C	T	*ORF1ab*					*	*
4925	G	T	*ORF1ab*	D1554Y	*				
5700	C	A	*ORF1ab*	A1812D	*	*		*	*
6317	C	T	*ORF1ab*	P2018S		*			
7070	G	T	*ORF1ab*	G2269C				*	
9246	C	T	*ORF1ab*	A2994V				*	
12469	C	T	*ORF1ab*			*			
14408	C	T	*ORF1ab*		*	*	*	*	*
15530	G	T	*ORF1ab*	V5089F					*
16887	C	T	*ORF1ab*	T5541I				*	
17325	G	A	*ORF1ab*	C5687Y		*			
17406	A	G	*ORF1ab*	D5714G					*
18877	C	T	*ORF1ab*				*		
19314	A	G	*ORF1ab*	H6350R				*	
19656	G	T	*ORF1ab*	R6464M					*
19810	A	G	*ORF1ab*					*	
20264	A	C	*ORF1ab*	N6667H			*		
20384	C	T	*ORF1ab*					*	
20647	C	T	*ORF1ab*				*		
21034	C	T	*ORF1ab*				*		
21513	C	T	*ORF1ab*	T7083I				*	
21786	G	T	*S*	G75V			*		
22329	C	T	*S*	S256L	*				
22585	T	G	*S*					*	
23031	T	C	*S*	F490S				*	
23403	A	G	*S*	D614G	*	*	*	*	*
24919	C	T	*S*					*	
24982	T	–T	*S*					*	*
25563	G	T	*ORF3a*	Q57H			*		
26735	C	T	*M*				*		
26924	A	G	*M*						*
27143	C	T	*M*		*				
27742	A	+A	*ORF7a*			*			
27827	G	T		*				
27986	T	A	*ORF8*						*
28183	G	T	*ORF8*	S97I			*		
28271	A	G		*				*
28277	T	C	*N*	S2P			*		
28280	G	T	*N*	D3Y		*			
28881	G	A	*N*	R203K		*		*	
28882	G	A	*N*			*		*	
28883	G	C	*N*	G204R		*		*	
29474	G	T	*N*	D401Y			*		

a Asterisks represent the presence of a mutation.

About 0.3 to 1.15 million reads were generated, with coverage in the range of 5,000 to 12,000×. Consensus sequences for each of the samples were generated using mpile-up in SAMtools v1.10 (6). The genomic GC content ranged from 38 to 40%, and the length of sequences ranged from 29,694 to 29,866 bp, covering 99.3 to 99.8% of the reference genome.

A phylogenetic analysis was conducted (7); the sequences were clustered using Augur v6.3.0 and aligned using MAFFT v7.471. Maximum likelihood trees were generated using IQ-TREE v1.6.12 and visualized using Auspice v2.0 (8) (Fig. 1). Four out of the five variants belonged to clade 20B, and one belonged to clade 20A. PANGOLIN v2.1.6 (www.github.com/cov-lineages/pangolin) was used to determine the lineages—two variants belonged to lineage B.1.1.306, and three variants belonged to lineages B.1.36, B.1.1.32, and B.1.1.281. All four lineages were previously associated with other Indian variants (https://cov-lineages.org/lineages). Sequencing of additional Indian viral variants in the future will be useful for understanding transmission, immune resistance, and vaccine efficacy in the population toward mitigation of a possible second wave of COVID-19 in India.

**FIG 1:** Phylogenetic analysis of SARS-CoV-2 genome sequences. Comparison of the five strains present in the study with 148 sequences from different parts of the Mumbai metropolitan region (through January 2021) were extracted from the GISAID database (https://www.gisaid.org/). Phylogenetic analysis was performed using the Augur v6.3.0 pipeline and visualized using Auspice v2.0, both developed by Nextstrain. The red dots indicate the five variants in the phylogenetic tree. Based on the Nextstrain nomenclature, four out of five variants (India/MH-CMP-19/2020, India/MH-CMP-30/2020, India/MH-CMP-34/2020, and India/MH-CMP-35/2020) belong to clade 20B, whereas one variant (India/MH-CMP-31/2020) belongs to clade 20A.

### Data availability.

The data from this study can be found under GISAID accession numbers EPI_ISL_779703, EPI_ISL_779705, EPI_ISL_779706, EPI_ISL_779708, and EPI_ISL_779710 (the sequences can be downloaded from GISAID at https://www.gisaid.org/); GenBank accession numbers MW645473, MW645474, MW645475, MW645476, and MW645477; SRA accession numbers SRR13892481, SRR13892480, SRR13892479, SRR13892478, and SRR13892477; and BioProject accession number PRJNA707397.
